# The Study on the Influence of Green Inclusive Leadership on Employee Green Behaviour

**DOI:** 10.1155/2022/5292184

**Published:** 2022-10-11

**Authors:** Dongmei Quan, Leyao Tian, Wenqi Qiu

**Affiliations:** School of Business, Qingdao university, Qingdao 266061, China

## Abstract

As a result of the implementation of the “double carbon” strategy, the issue of how to encourage green behaviour has become a prominent one in society. According to the cognitive-affective processing system theory, this study constructs two paths through which green inclusive leadership influences employee green behaviours: the cognitive pathway mediated by pro-environmental goals clarity and the affective way mediated by green organization identification. Data analysis of 372 employees in chemical enterprises reveals that first, employees' perception of green inclusive leadership positively affects employee green behaviour; second, green inclusive leadership enhances employee awareness of environmental goals and green organization identification so that employees are more likely to behave environmentally; furthermore, green HRM practices positively moderate the relationship between green inclusive leadership and pro-environmental goals clarity, as well as positively moderate the relationship between green inclusive leadership and green organization identification. This study aims to provide theoretical and practical insight into how to promote the green development of organizations from the perspective of leadership style to facilitate green development.

## 1. Introduction

The world is pumping about 51 billion tons of greenhouse gases into the atmosphere every year, which is making the phenomenon of global warming increasingly serious, along with the attendant environmental problems such as rising sea levels, rising Arctic temperatures, and natural disasters. To avoid climate catastrophe, humans need to stop pumping greenhouse gases into the atmosphere and achieve zero emissions. The country has implemented the “double carbon” strategy of carbon peak and carbon neutrality, which calls for enterprises to reduce carbon emissions and lead enterprises in sustainable management practices. To respond to the national double-carbon policy, academia and entrepreneurs are focusing on what kind of leadership mode enterprises should adopt to encourage employees to take the initiative in green behaviour. A new leadership style has been proposed called green inclusive leadership [1]. In contrast with other leadership styles, this style is characterized by an openness to employee suggestions for green ideas, a willingness to discuss with employees the organization's environmental goals, and an acceptance of employees' input regarding ecological challenges. A recent study shows that green inclusive leadership can create a green psychological atmosphere and increase engagement with green work [1]. It remains unclear, however, whether green inclusive leadership will influence employees' green behaviour and through what mechanism. We discuss the above problems to provide reference significance to enterprises promoting green behaviours among their employees.

Previous studies have explored the relationship between green leadership and employees' green behaviour, but the mechanism of how green inclusive leadership affects employees' green behaviour has not been examined. Cognitive-affective system processing theory suggests that a person's cognitive response and affective response are intertwined and affect each other simultaneously. By influencing the employee's cognition and affection, the leader can influence the employee's behaviour. Currently, studies primarily focus on affective factors, such as employees' environmental responsibility [2] and positive emotion [3], ignoring the influence of cognition on employee behaviour. The basic concept of cognitive-affective processing system theory holds that behaviour is determined by how cognition and affection interact. Therefore, we believe that, on the one hand, green inclusive leadership cognitively conveys the environmental goals of the organization and expectations for environmental performance to employees. Employees will be more explicit about the objectives. They will pay better attention to the organization's environmental objectives, aligning their behaviour towards its goals, and encouraging employees to behave greenly. On the other hand, environmental protection and green values are conveyed emotionally to employees through green inclusive leadership. Employees will demonstrate green behaviours if the organization's values are aligned with their own. We explored how green inclusive leadership influences employees' green behaviour by introducing two cognitive and affective units of proenvironmental goal clarity and green organization identification as critical cognitive and affective units between green inclusive leadership and green behaviour [4]. Therefore, proenvironmental goal clarity and green organization identification may mediate between green inclusive leadership and employee green behaviour.

Moreover, it is not just the leader who has the power to influence employees. Human resource management systems are all responsible for recruiting, selecting, evaluating, and promoting employees, so policies and measures implemented by the human resource management department can also influence and alter employees' working attitudes and behaviours. It is more likely that employees will accept the green concept conveyed by the organization when the human resource department makes corresponding green policies and requires them to pay attention to sustainable and green development. HRM measures in green management are called green HRM practices, specifically incorporating environmental protection and green sustainability concepts into various HRM modules [5]. Employees will be more likely to engage in green behaviours if they know that a high-level green human resource management practices are being implemented in the organization. Alternatively, if the organization does not implement green human resource management practices, employees will not pay attention to green behaviour, resulting in lower performance. We incorporated green human resource management practice as a moderating variable in our theoretical model based on social information processing theory [6]. We tested whether green human resource management practice moderates the relationship between cognitive and affective units and green inclusive leadership. Examine what boundary conditions green inclusive leadership requires.

Three aspects contribute mainly to the research contribution of this paper. Firstly, from the perspective of “cognition-affection,” the influence mechanism of green inclusive leadership on employees' green behaviour is discussed, expanding the research content of green inclusive leadership and breaking from previous limitations based on the single emotional perspective. We proposed and tested the dual mediating effect of proenvironmental goal clarity and green organization identification, revealing how cognitive and affective factors influence green inclusive leadership and green employee behaviour. Secondly, few studies have simultaneously examined the impact of organizational human resource management practices and leadership behaviour. It indicates that green human resource management practices have a moderating effect on individual behaviour, enriching the research on the relationship between human resource management and individual behaviour, as well as expanding the research on the context of green inclusive leadership and its boundary conditions. Thirdly, employee green behaviour is crucial in improving their environmental performance for organizations to achieve environmental goals. This paper enhances research on influencing factors of green behaviour among employees. A cognitive-affective model has rarely been used to study employee green behaviour. In this study, cognitive and affective approaches were used to explore the antecedent effects of green inclusive leadership on employee environmental goal clarity and green organization identification, enhancing research on leadership and individual behaviour.

## 2. Research Hypothesis

### 2.1. Green Inclusive Leadership and Employee Green Behaviour

A green inclusive leadership style involves interacting with employees to achieve environmental protection and cleanliness organizational goals [1]. Openness, effectiveness, and accessibility are the characteristics of this leadership style. The organization's leaders are open to new green ideas and willing to discuss environmental goals and consult on environmental issues. Employee green behaviour refers to the behaviours of employees in the workplace that support environmental sustainability [7], such as turning off lights, providing environmental protection advice, or participating in environmental protection projects. In the process of work, the leader is the core of moral guidance for the members of the organization. The employees will be more actively committed to the green behaviour of the organization when the leader supports the internal environmental protection work of the organization, takes the initiative to guide them, and tolerates opinions and suggestions that differ from their own [8].

According to social information processing theory, people's attitudes and behaviours are influenced by the environment around them. How employees process and analyze information and cues influences work attitudes and behaviours. The concept of green, environmental protection, and sustainability is carried out in the interaction between green inclusive leaders and their subordinates. Employees will store such information in their memory when they receive it. When relevant events require judgment and further action, employees will retrieve information about environmental protection and sustainability in their memory and make judgments and inferences based on it. Leaders who support employees' environmental behaviours will give them fundamental guarantees that they will participate in proenvironmental behaviours and develop environmental initiatives. These behaviours will influence employees psychologically, resulting in an internal motivation to engage in green behaviour [9].

Researchers have found that green inclusive leadership affects employees' green psychological atmosphere [1] and then promotes green behaviours. Leadership that is inclusive sets an example for employees, sees everyone as equal, and recognizes their efforts, all while maintaining an open view of individuals' differences with their different opinions and suggestions [10]. As a result of this psychological state, employees are more likely to express their ideas and more inclined to work towards the organization's goals. Supporting and encouraging employees' green behaviours in their daily work will likely increase their green behaviours. Accordingly, the following hypothesis is proposed:

(H1) : green inclusive leadership positively influences employees' green behaviour.

### 2.2. The Mediating Effect of Pro-environmental Goal Clarity and Green Organization Identification

Cognitive-affective processing system theory proposes that employees are rational and sensual organisms. Cognitive-affective units interact with events that people encounter and ultimately determine their behaviours. Therefore, employees' green behaviours are influenced by their cognition and affection. On the one hand, as employees become familiar with the organization's expectations for environmental performance and goals, they will become more cognizant of environmental protection and green behaviours. On the other hand, employees will be infected and influenced when the organization has a green atmosphere and conveys the sentiment of being green and sustainable, which will lead them to develop a green psychological atmosphere and act greenly. Cognition-affective system theory provides a good perspective on how leadership contributes to employee green behaviour. In particular, green inclusive leadership affects employees' green behaviours cognitively and affectively.

In one sense, proenvironmental goal clarity is reasonable as a measure of cognitive response. The characteristics of cognitive responses suggest that when individuals process information from the perspective of analysis, they will carefully observe things and evaluate them logically and causally [11]. The clarity of environmental goals reflects the understanding and clarity of individual employees' green and environmental goals [12], which should be determined objectively. As a measure of affective reaction, green organization identification is reasonable. An organization's leadership style reflects its culture, while green inclusive leadership reflects its environmental and green values. When employees reflect on the organization's green culture, they will identify with the green organization [13] and then show green behaviour.

Using cognitive-affective system processing theory, social information processing theory, and organizational identity theory, we also reveal how green inclusive leadership affects employees' green behaviour cognitively and affectively.

#### 2.2.1. The Mediating Effect of Pro-environmental Goal Clarity

Employees can become more aware of the external environment by being exposed to organizational goals. A difference in understanding and acceptance of organizational goals will lead to varying clarity of goals and cognitive differences [14]. According to the social information processing theory, green inclusive leaders are one of the main sources of information for employees to know and understand the organization's environmental goals, providing them with information about the organization's environmental behaviour, and strengthening employees' awareness of the organization's environmental goals. On the one hand, within the organization leadership style for the green inclusive leadership, staff and leaders will be in benign interactions and communication, and leaders will be tolerant of employee questions and made mistakes. They will accept suggestions and comments that differ from their own. In this case, employees are more likely to accept the organization's objectives, further clarifying organizational goals. On the other hand, green inclusive leadership communicates environmental goals to employees, who will accept their green and sustainable ideas and understand that environmental protection is also the work goal of the organization's members, making employees' environmental goals clear.

Goal clarity refers to a person's understanding of job objectives and responsibilities [15]. The goal-setting theory suggests that clear work goals can help individuals make good decisions, make them more focused, and help them achieve their goals [16]. A clear and specific perception of the organization's goals will lead to employees understanding of their own goals. The clarity of environmental objectives reflects that employees can clearly and accurately understand the environmental objectives of the organization, as well as the clarity of individual employees' environmental protection objectives and responsibilities. Employees with a high definition of environmental goals clearly understand that going green is one of the goals of the organization members, for their responsibilities and organization has a more precise and accurate cognition of their expectations, thereby reducing behaviour blindness, improving employees' self-control ability, motivating them to pursue their goals and perseverance, pursuing an environment consistent with the organization's environmental goals, and exhibiting more green behaviour.

As a result of green inclusive leadership, employees can be better informed about the organization's environmental goals, improve their clarity of environmental goals, have a clearer understanding of their environmental responsibilities, reduce blindness to actions, and act more environmentally friendly. Based on this, we put forward the following hypothesis:

(H2) : proenvironmental goal clarity mediates the relationship between green inclusive leadership and employee green behaviour.

#### 2.2.2. The Mediating Effect of Green Organization Identification

Green organization identification is a model established by the organizational members to identify environmental management and green innovation to give meaning to environmental protection behaviour [17]. Employees with organization identification are emotionally connected to the organization. The words and actions of leaders profoundly impact organizational members, so they contribute to employees' identification with the organization [18]. Identifying with green organizations results from employees' feelings about environmental protection and sustainable development conveyed by green inclusive leadership. Employees will commit to green behaviours more actively if they are emotionally consistent. Employees' organizational identity is significantly affected by their organization's image [19]. An excellent organizational image is essential for employees to form an organizational identity, and the management style affects how the organization shapes its image. The leadership style of its leaders may shape an organization's image. Employees can enhance their green organizational identity by working in an environment that promotes environmental protection and sustainability. Organizational climate, however, significantly impacts organization identification [20]. An excellent organizational climate helps employees form more positive perceptions of the organization. They are incorporating green environmental protection into the organizational climate resulting from green inclusive leadership. Meanwhile, inclusive leadership fosters a harmonious atmosphere within the organization and contributes to employees' identification with the organization as green. Organizational identity is also significantly influenced by organizational culture [21]. The role of leaders in influencing organizational culture is to give meaning to employees and to build meaning for them. An organization's green and environmental protection culture can be shaped by green inclusive leadership. Employees should then have a green identification in their organization.

According to some studies, identifying an organization as green may improve its environmentally friendly behaviour [22]. According to the organizational identity theory, persistence in pursuing goals can be affected by organizational identity. In general, the more employees identify with an organization, and the more enthusiastic they are about taking action. Alternatively, employees with a solid organizational identity will identify more with their organization and evaluate it more highly, improving its image and quality through positive behaviours. Employees' emotional connection to how an organization handles environmental issues encourages them to consider environmental protection as one of their responsibilities and exhibit green behaviour as a result.

Having green inclusive leadership will lead to a green and environmentally friendly organization image, create a green organizational atmosphere, shape a green and sustainable organizational culture, and enhance employees' sense of belonging to a green organization. Employees with high green organization identification will take more positive actions to protect the organization, leading to more green behaviours. Based on this, the following hypothesis is proposed:

(H3) : green organization identification plays a mediating role between green inclusive leadership and employee green behaviour.

### 2.3. The Moderating Effect of Green Human Resource Management Practice

As leaders and HRM practices in the organization affect employee attitudes and behaviours, we introduce green HRM practices into the research model. For organizations to carry out green management, green human resource management practice is a method, which is to say, the human resource management of organizations carries out green management, standardizing the management of employees' green behaviours on a system and policy level [23]. Among the practical dimensions of green human resource management are recruitment and training, compensation design, performance appraisal, and employee participation [24].

In organizations with green and inclusive leadership styles, employees perceive clearer and more accurate environmental goals and behave more sustainably. The role of human resource management is to connect the organization with its employees. The organization uses it to conduct training, compensation design, and performance appraisals for its employees. The organization provides the employees with corresponding environmental protection clues, conveys the organization's concept and goal, and can improve their understanding of the environmental protection goal. During the recruitment process, green human resource management focuses on selecting employees who align with the environmental values of the organization. Since these employees are more convinced of the green inclusive leadership style, they can help clarify environmental objectives. The training session promotes environmental knowledge and skills among employees. In this case, it makes sense to deepen employees' understanding of green inclusive leadership so they realize the organization values green goals and thus improve environmental goals' clarity. In the process of employee performance appraisal and salary design, tying green environmental responsibility to employee performance and salary will promote the application and practice of green environmental protection and sustainable concepts advocated by green inclusive leadership and motivate employees who perform green environmental responsibility with salary. As a result, employees will be more aware of the organization's environmental goals. Green and inclusive leadership styles can encourage employees to set clear environmental goals within an organization. At this time, if the organization implements green human resources management practices, from staff recruitment, training, compensation design, performance appraisal, and employee involvement, employees will provide clues to their organization's commitment to preserving the environment. Both leadership and management systems provide employees with environmental cues that emphasize the importance of environmental protection. According to the cued coherence theory [25], this further enhances employees' perception of the organization's environmental goals and clarifies employees' environmental goals.

As mentioned above, when the internal leadership style of an organization is green and inclusive, it will create a green corporate image, organizational atmosphere, and organizational culture, and employees will generate more green organization identification, which will lead to green behaviour. As a result of green human resource management practices, leaders conduct green management among employees, and employees will have more trust and understanding of green inclusive leadership and form the same pursuits of green values as the organization, resulting in higher recognition of green organizations. During recruitment, green human resource management practices emphasize selecting employees with good environmental awareness [26]. They are more likely to identify with green organizations because they are more likely to identify with green inclusive leadership styles. The training process will include attention to the green culture and concept of the enterprise, strengthening the understanding of green inclusive leadership of employees, which will lead to green organization identification. As part of employee performance appraisals and salary designs, green environmental responsibility should be incorporated into employee salaries so that employees know the organization's sustainability expectations. Employees are more likely to identify their organization as green when exposed to green inclusive leadership practices and concepts. When employees recognize the significance of the organization's green human resource management practices, the impact of green inclusive leadership on employees will be enhanced, and employees will identify more with green organizations.

Following the social information processing theory, employees will have more trust in green inclusive leadership when they experience the implementation of green human resource management practices, which leads to a clearer understanding of employees' environmental goals and a better ability to identify green organizations. Based on this, the following hypotheses are proposed:

(H4) : green human resource management practices positively modify the relationship between the green inclusive leadership and the proenvironmental goal clarity.
(H5) : green human resource management practices positively modify the relationship between the green inclusive leadership and the green organization identification.

To sum up, the dual-mediation theoretical model established in this study is shown in Figure 1.

## 3. Research Methods

### 3.1. Data Collection and Research Samples

The study was conducted online and field research for six months, from November 2021 to April 2022. This paper aims to examine green behaviour in five large chemical enterprises in Qingdao, Beijing, and other places since green behaviour is prevalent in chemical enterprises. An adapted two-stage survey method was used in this study to reduce the influence of common method bias. A survey was conducted twice, with a three-month interval between each questionnaire. Employee perceptions of green inclusive leadership, green HRM practices, and control variables were included in the first stage survey. In contrast, the second stage survey included employees' proenvironmental goals clarity, green organization identification, and employee green behaviour.

The survey purpose was explained to the enterprise in advance, and the survey results were kept confidential. As a condition of receiving the research results, we promised not to use them for any other purpose. A field survey was conducted for the first survey. A numbered questionnaire was distributed to the employees through the human resource management department, and the human resource management department and researchers recorded the employee numbers. The total number of questionnaires distributed this time was 500. Employees who answered the questionnaires effectively in the first survey were selected for the second survey three months later. We distributed 430 questionnaires to employees online. In order to match the information of the two surveys, we also numbered them.

Ultimately, this survey collected effective data on 372 employees, resulting in a recovery rate of 74.4%. In the sample analysis, males accounted for 52.2%, and females accounted for 47.8%; (2) 18.3% of the employees are under 25 years old, 44.3% are between 26 and 35 years old, 27.7% are between 36 and 45 years old, and 9.7% are over 46; (3)18.3% of employees have a high school degree or below, 28.2% have a college degree, 44.4% have a bachelor's degree, and 9.1% have a master's degree or above. (4) 21.2% of the employees have worked for less than one year, 30.6% for one to three years, 32.3% for four to six years, and 15.9% for more than seven years.

### 3.2. Research Tools

All variables in this study were measured using the developed mature scale. All questions were translated and back-translated to avoid misunderstandings due to cultural differences. All the questionnaires were evaluated by a Likert 7-point scale, where 1 means “strongly disagree” and 7 means “strongly agree.” Specific variable items are shown in Table 1.

Green Inclusive Leadership (GIL): a 3-question scale developed by Bhutto et al. [1]. In this study, the reliability coefficient of the scale was 0.887.

Proenvironmental Goal Clarity (PGC): a 5-question scale developed by Liang et al. [18]. In this study, the reliability coefficient of the scale was 0.822.

Green Organization Identification (GOI): a 6-item scale developed by Chen [27]. In this study, the reliability coefficient of the scale was 0.883.

Employee Green Behaviour (EGB): a 7-item scale developed by Robertson and Barling [28]. In this study, the reliability coefficient of the scale was 0.858.

Green Human Resource Management Practices (GHRM): the scale developed by Ogberbu et al. [29] is divided into three dimensions: green recruitment and selection, green performance and compensation, and green training participation and development. According to the Chinese context, this study selected 14 items on the scale. Employees select the perceived green HRM practices according to the actual situation. In this study, the reliability coefficient of the scale was 0.910.

The employees' age, gender, and education level are used as control variables. Furthermore, since the employee's working years will affect their working behaviour and performance, the employee's working years are also included as a control variable.

## 4. Data Analysis and Results

### 4.1. Confirmatory Factor Analysis

To determine the validity of the variables, we conducted a confirmatory factor analysis on five key variables, such as “green inclusive leadership,” “proenvironmental goals clarity,” “green organization identification,” “green human resource management practice,” and “employee green behaviour.” Table 2 compares the fitting results of the five-factor, four-factor, three-factor, two-factor, and one-factor models. There is a significant improvement in the relevant effect of the five-factor model (*χ*^2^/df = 2.01, RMSEA = 0.05, TLI = 0.90, CFI = 0.91, SRMR = 0.045), and each index is significantly better than the other four models. These data indicate that the five variables in this study have good discriminant validity.

### 4.2. Common Method Bias Analysis

An anonymous questionnaire was filled out during the data collection stage, and a two-stage collection method was used. To reduce the homologous variance problem, we promised employees before completing the data collected by this questionnaire that the research results would not be used for any other purpose than scientific research before completing the questionnaire. To assess the severity of the common method bias in the study data, the Harman single factor test [30] was used. The principal component factor analysis was conducted on all items of the five main variables. In the test results, 23.596% of the variation was explained by the first principal component and 68.235% by the cumulative component, which did not account for 40% of the total variance. The KMO was 0.869, and the Bartlett was 13061.083, which were significant at the 0.001 level. Also, all the fit indices for the five-factor model are within the reference range. In contrast, all of the fit indices for the one-factor model are outside the reference range, indicating that the fitting degree of the research data is good to some extent. As a result, this study does not exhibit any homologous severe variance bias.

### 4.3. Descriptive Statistical Analysis

Each variable's mean, standard deviation, and correlation coefficient are shown in Table 3. Green inclusive leadership is positively correlated with the proenvironmental goals clarity, green organization identification, and employee green behaviour (*r* = 0.437, *P* < 0.01; *r* = 0.291, *P* < 0.01; *r* = 0.263, *P* < 0.01); the green behaviour of employees was positively correlated with the proenvironmental goals clarity and green organization identification (*r* = 0.378, *P* < 0.01; *r* = 0.346, *P* < 0.01), which provided a preliminary basis for further exploring the relationship between variables.

### 4.4. Hypothesis Testing

#### 4.4.1. Main Effect Test

This study uses five nested models to examine the simultaneous mediating effects of proenvironmental goals clarity and green organization identification. The results are shown in Table 4. Using M1, a partial mediation model, we explore the direct impact of green inclusive leadership on employee green behaviour and the simultaneous mediating effect of proenvironmental goals clarity and green organization identification. The M2 model deleted the direct path and only included the full mediation model that dictates that proenvironmental goals clarity and green organization identification indirectly influence employee green behaviour. The M3 model measures the influence of green inclusive leadership on the proenvironmental goals clarity of employees after controlling for green organization identification. Employee green behaviour is directly affected by green inclusive leadership and indirectly by green organization identification. M4 is a partial mediation model in which proenvironmental goals clarity is the mediating variable after controlling for green inclusive leadership's influence on employees' green organization identification. Employee green behaviour is directly influenced by green inclusive leadership and indirectly influenced by proenvironmental goals. The M5 model is a direct action model. After controlling green inclusive leadership for its influence on green organization identification and proenvironmental goals clarity, it is examined for its direct impact on employee green behaviours. Gender, age, education, and tenure are used as control variables in the five models.

Based on the test results of M5, it is demonstrated that, after controlling the influence of green inclusive leadership on the proenvironmental goals clarity and the green organization identification, green inclusive leadership significantly affects employee green behaviour (*β* = 0.212, *P* < 0.001), proving hypothesis 1. Green inclusive leadership also had a significant impact on proenvironmental goals clarity (*β* = 0.368, *P* < 0.001) and green organization identification (*β* = 0.216, *P* < 0.001). After adding two mediating variables, M1 was obtained. At this time, compared with the test results of M5, the impact of green inclusive leadership on employee green behaviour was no longer significant (*β* = 0.010, *P* > 0.05). However, the proenvironmental goals clarity had a significant positive impact on employee green behaviour (*β* = 0.386, *P* < 0.001). There was a significant positive relationship between green organization identification and employee green behaviour (*β* = 0.281, *P* < 0.001). A significant relationship between employee green behaviour and green inclusive leadership was found when comparing M3 with M5 when M3 offered only green organization identification. A comparison between M4 and M5 showed that only when the proenvironmental goals clarity was introduced into M4, the effect on the green behaviour of employees was not significant (*β* = 0.072, *P* > 0.05). Furthermore, the two mediating variables had significant effects on the dependent variable. There was a standardized path coefficient of 0.281 (*P* < 0.001) between green organization identification and employee green behaviour in M3 and 0.382 (*P* < 0.001) between proenvironmental goals clarity and employee green behaviour in M4. In the above model, the two mediating variables play a synchronous mediating role in the relationship between green inclusive leadership and employee green behaviour.

The analysis results in Table 4 show that the cognitive and affective mediating variables fully mediate the relationship between green inclusive leadership and employee green behaviour, which shows a better fit than when only the cognitive path or emotional path is considered. According to this paper, M2 was the most complete and had the highest reasonable degree of the five structural equation models, so M2 was selected as the final model.

#### 4.4.2. Mediating Effect Test

This study used the Hayes' Process program and Bootstrap method to estimate and test the mediating effect. A Bootstrap sample is run 5000 times, and the results are presented in Table 5. There is an indirect effect of proenvironmental goals clarity between the green inclusive leadership and the employee green behaviour of 0.141, 95% CI is 0.071, 0.238; and the confidence interval does not include 0. Hypothesis 2 is therefore confirmed. An indirect effect of green organization identification on employee green behaviour is 0.062, 95% CI is 0.026, 0.114; and the confidence interval does not include zero. It confirms hypothesis 3. The mediating effects of the two mediators were compared and tested using a double-mediation comparison model. The estimated value was 0.079, 95% CI was -0.002, 0.188; and the confidence interval included zero, which indicates that the two mediators have the same indirect effect status between green inclusive leadership and employee green behaviour. That is, they play an equally significant role.

#### 4.4.3. Moderating Effect Test

To test the moderating effect in this study, we used hierarchical regression analysis, and the results are shown in Table 6. We standardized green inclusive leadership and green human resource management practices to avoid multicollinearity.

Table 6 shows that the green inclusive leadership practices and the green human resource management practices significantly influence employee proenvironmental goals clarity (*β* = 0.126, P < 0.01). As found by T1, T2, and T3, after including green inclusive leadership, green human resource management practices, and their interaction terms, the overall explanatory quantity R2 of the model significantly increased, suggesting that green human resource management practices positively moderated the relationship between the green inclusive leadership and the proenvironmental goals clarity. Therefore, hypothesis 4 is true. Interaction between green inclusive leadership and green human resource management practices significantly enhanced employees' green organization identification(*β* = 0.162, *P* < 0.001). After incorporating green inclusive leadership, green human resource management practices, and their interaction terms, the overall explanatory quantity R^2^ of the model significantly improved. Accordingly, green human resource management practices positively regulate the relationship between green inclusive leadership and green organization identification, which confirms hypothesis 5.

To clarify the impact of green human resource management practices, Figure 2 shows the difference in the impact of green inclusive leadership on employee green behaviours under different degrees of green human resource management practices, with one standard deviation higher than and one standard deviation lower than the mean value of green human resource management practices. According to Figure 2, the more green human resource management practices, the stronger the impact of green inclusive leadership on proenvironmental goals clarity and green organization identification; conversely, the weaker. As can be seen, green human resource management practices have a moderated effect.

## 5. Conclusion and Discussion

### 5.1. Research Conclusions

The study examined 372 valid data samples based on the cognitive-affection processing system framework. It came to relevant conclusions about green inclusive leadership, proenvironmental goals clarity, green organizations identification, implementation of green human resources management practices, and employee green behaviour. Based on the results, we can conclude that firstly, a green inclusive leadership strategy can significantly increase the green behaviour of employees; secondly, environmental goals clarity and green organization identification play an integral role in mediating between green inclusive leadership and employee green behaviour; furthermore, green human resource management practices moderate the impact of green inclusive leadership on the identification of green organizations and the clarity of environmental goals.

### 5.2. Implications for Practices

Using the cognitive-affective processing system framework, we examine the relationship between green inclusive leadership and employees' green behaviour and draw the following implications for management practice:

- Enterprises must give the promotion effect of green inclusive leadership on employees' green behaviours a high priority. To be specific, the enterprise should be planned and targeted to develop green inclusive leadership, improve leadership's environmental protection knowledge and skills, establish green leadership, environmental protection, sustainable ideas, and concepts, to allow leaders to accept differences and open to green concepts, and actively promote green inclusive leadership. Furthermore, enterprise leaders should improve their interaction with employees on a two-way basis. As part of the communication process with employees, they should respect and acknowledge the efforts and contributions of each employee in environmental protection and encourage employees to express their opinions and suggestions
- Besides attaching importance to inclusive green leadership, enterprises need to adopt and implement green human resource management practices so that employees' green behaviour can be more effectively promoted and the organization's sustainable development can be promoted. Specifically, relying only on the leader's leadership style for management has limits, as ensuring that the leader's values convince every employee is challenging. As a result, enterprises should establish a set of standardized rules and regulations related to green management, integrate environmental protection into each human resource management module, and provide institutional guarantees for leaders' green management behaviours. Implement a sound green human resource management system
- Enterprises should emphasize employees' clear cognition and understanding of corporate environmental goals, as well as employees' green identification within the organization, in applying green inclusive leadership and green human resource management. Employees should be informed of the company's expectations for environmental goals and the environmental responsibilities they should take to incorporate them into their job duties. The organization should also establish a green consciousness and correct environmental concept among its employees, make them consistent with its environmental protection concept, let employees participate in the work to protect the environment, and encourage them to behave in a greener way
- In addition to the management of enterprises, employees should also be inspired. Employees should pay attention to the importance of environmental goals in the workplace or in unusual places, actively cooperate with the initiative of green inclusive leadership, take the initiative to comply with the relevant regulations put forward by green human resource management, and take the initiative to make green behaviours. Employees should clearly realize that this is not only the behaviour that the enterprise values, but also the green behaviour that is beneficial to the country and even the world

### 5.3. Research Limitations and Further Research Directions

Due to the conditions, this paper still has the following shortcomings: as a first step, we only explore the influence mechanism of green inclusive leadership on employee individual behaviour and explore the influence of leadership on employee behaviour from the perspective of individual perception. Insufficient research has been conducted on other levels and across levels. Examining the influence mechanism at the team and organizational levels can further expand the research in this area.

Additionally, based on the research data, the questionnaire was issued with certain limitations. In the future, research should expand the scope, provide prosperous research industries and regions, increase the number of representative studies, and make research conclusions more universal and extensible.

Furthermore, although this paper uses two-node questionnaire surveys, the data are still cross-sectional. Therefore, in the future, it can use longitudinal research methods to test the impact of green inclusive leadership on employee behaviour and examine the dynamic effect of green inclusive leadership on employees' green behaviours, improving the study's accuracy.

## Figures and Tables

**Figure 1:** Mechanism of the role of green inclusive leadership on employee green behaviour.

**Figure 2:** Reconciliation path diagram.

**Table 1:** Variable items.

	Items
GIL	(1) The leadership in the organization is willing to discuss with employees environmental goals at work and new green ways to achieve these goals (2) Employees can consult with leaders in the organization about environmental issues at work (3) The organization's leaders are willing to listen to and deal with employees' requests related to environmental issues at work

PGC	(1) I am clear about my environmental responsibilities (2) I have a clear understanding of my environmental objectives (3) I am clear about the expected outcomes of my environmental activities (4) I am clear about which environmental activities will be positively evaluated (5) I am aware of the link between my environmental activities and the overall objectives of my department

GOI	(1) Employees are very aware of the company's environmental management and conservation history (2) Employees are proud of the company's environmental goals and mission (3) Employees believe that the company has achieved an important position in environmental management and protection (4) Employees believe that the company has established a clear set of environmental objectives and mission (5) Employees are aware of the company's environmental traditions and culture (6) Employees strongly agree with the company's actions in environmental management and protection

EGB	(1) I will print on both sides when possible (2) I will put compostable items in the compost bin (3) I will put recyclable materials in the recyclable bin (4) I will bring reusable tableware to work (5) I turn off lights that are not in use (6) I will participate in environmental projects (7) I would make suggestions about environmental practices to improve the environmental performance of the organization

GHRM	(1) The company focuses on recruiting and selecting employees who are environmentally conscious and have environmental knowledge and skills (2) The company attaches importance to the candidate's attitude and concern for environmental protection in the recruitment process (3) The company carefully design interview questions to examine candidates' attitudes, knowledge, skills, and concern for the environment (4) The environmental objectives set by the company's management can be implemented (5) The company incorporates environmental performance indicators into the evaluation system of managers' work (6) The company includes environmental performance indicators in the evaluation system of employees (7) The company gives nonmonetary rewards to employees who achieve environmental performance targets (8) The company will adjust employee compensation based on environmental performance (9) Employees are well-recognized and rewarded for their environmental initiatives (10) The company provides training for employees in environmental protection-related knowledge and skills (11) The company provides training for managers in environmental protection-related knowledge and skills (12) The company has a job description that describes its environmental responsibilities (13) Company members participate in discussions on environmental issues (14) After receiving training in environmental protection skills, company members can apply green knowledge in their daily work

**Table 2:** Confirmatory factor analysis.

Model	*χ* ^2^	Df	*χ* ^2^/df	RMSEA	TLI	CFI	SRMR
Five-factor model	1102.76	550	2.01	0.052	0.90	0.91	0.045
Four-factor model	1728.86	554	3.12	0.076	0.79	0.80	0.084
Three-factor model	2914.76	557	5.23	0.107	0.58	0.60	0.166
Two-factor model	3571.73	559	6.39	0.121	0.46	0.50	0.168
One-factor model	4472.25	560	7.99	0.137	0.31	0.35	0.174

Note: five-factor model (green inclusive leadership; proenvironmental goals clarity; green organization identification; green human resource management practice; and employee green behaviour); four-factor model (green inclusive leadership; integration of proenvironmental goals clarity and green organization identification; green human resource management practice; and employee green behaviour); three-factor model (green inclusive leadership; integration of proenvironmental goals clarity, green organization identification and green human resource management practices; and employee green behaviour); two-factor model (integration of green inclusive leadership, proenvironmental goals clarity, green organization identification and green human resource management practices; and employee green behaviour); single-factor model: all variables are combined.

**Table 3:** Mean, SD, and correlations coefficient of the studied variables.

Variables	M	SD	1	2	3	4	5	6	7	8
1 Gender	1.48	0.52	一							
2 Age	2.29	0.88	-0.077	一						
3 Education	2.44	0.88	0.052	-0.015	一					
4 Tenture	2.43	1.00	0.008	0.131^∗∗^	-0.011	一				
5 GIL	4.25	1.50	-0.037	0.020	-0.012	-0.002	一			
6 PGC	4.71	1.13	0.096	0.016	-0.006	-0.010	0.437^∗∗^	一		
7 GOI	5.08	1.05	0.069	0.025	-0.055	-0.045	0.291^∗∗^	0.207^∗∗^	一	
8 EGB	4.54	1.05	-0.006	0.041	0.004	-0.045	0.263^∗∗^	0.378^∗∗^	0.346^∗∗^	一
9 GHRM	5.52	0.92	0.070	-0.033	0.102	0.045	0.197^∗∗^	0.003	0.024	0.043

Note: *n* = 372, ^∗^*P* < 0.05, ^∗∗^*P* < 0.01, ^∗∗∗^P < 0.001.

**Table 4:** Comparison between structural equation models.

	M1 GIL⟶PGC⟶EGB GIL⟶EGB GIL⟶GOI⟶EGB	M2 GIL⟶PGC⟶EGB GIL⟶GOI⟶EGB	M3 GIL⟶PGC GIL⟶EGB GIL⟶GOI⟶EGB	M4 GIL⟶PGC⟶EGB GIL⟶EGB GIL⟶GOI	M5 GIL⟶PGC GIL⟶EGB GIL⟶GOI
GIL⟶PGC	0.524^∗∗∗^	0.371^∗∗∗^	0.370^∗∗∗^	0.370^∗∗∗^	0.368^∗∗∗^
PGC⟶EGB	0.386^∗∗∗^	0.390^∗∗∗^		0.382^∗∗∗^	
GIL⟶EGB	0.010		0.151^∗∗∗^	0.072	0.212^∗∗∗^
GIL⟶GOI	0.220^∗∗∗^	0.220^∗∗∗^	0.220^∗∗∗^	0.220^∗∗∗^	0.216^∗∗∗^
GOI⟶EGB	0.281^∗∗∗^	0.284^∗∗∗^	0.281^∗∗∗^		
*χ* ^2^/*d*f	1.682	1.673	1.679	1.679	1.667
RMSEA	0.043	0.043	0.043	0.043	0.042
CFI	0.964	0.965	0.965	0.964	0.965
TLI	0.959	0.960	0.960	0.959	0.960
SRMR	0.041	0.041	0.041	0.041	0.036

**Table 5:** Comparison of mediating effect and double mediating effect.

	Estimate	Standard deviation	Lower limits	Upper limits
GIL⟶PGC⟶EGB (a)	0.141	0.043	0.071	0.238
GIL⟶GOI⟶EGB (b)	0.062	0.023	0.026	0.114
(a, b)	0.079	0.049	-0.002	0.188

**Table 6:** Results of the moderating effect analysis.

Variable	PGC			GOI		
	T1	T2	T3	T4	T5	T6
Gender	0.098	0.120^∗∗^	0.132^∗∗∗^	0.075	0.088	0.092
Age	0.025	0.013	0.014	0.037	0.030	0.031
Education	-0.011	0.003	0.001	-0.058	-0.052	-0.056
Tenure	-0.014	-0.007	-0.012	-0.051	-0.048	-0.055
GIL		0.460^∗∗∗^	0.453^∗∗∗^		0.300^∗∗∗^	0.291^∗∗∗^
GHRM		-0.087	-0.044		-0.033	0.021
GIL × GHRM			0.126^∗∗∗^			0.162^∗∗∗^

R^2	0.010	0.213	0.226	0.012	0.098	0.121
F	0.924	15.219^∗∗∗^	16.789 ^∗∗∗^	1.071	6.634^∗∗∗^	7.181^∗∗∗^
△R^2^	0.010	0.203	0.013	0.012	0.086	0.023

## Data Availability

The experimental data used to support the findings of this study are available from the corresponding author upon request.
